# *Bordetella pertussis* and *Bordetella bronchiseptica* filamentous hemagglutinins are processed at different sites

**DOI:** 10.1002/2211-5463.12474

**Published:** 2018-06-20

**Authors:** David Jurnecka, Petr Man, Peter Sebo, Ladislav Bumba

**Affiliations:** ^1^ Laboratory of Molecular Biology of Bacterial Pathogens Institute of Microbiology Czech Academy of Sciences Prague 4 Czech Republic; ^2^ Department of Biochemistry Faculty of Science Charles University in Prague Prague 2 Czech Republic; ^3^ BioCeV ‐ Institute of Microbiology of the Czech Academy of Sciences Vestec Czech Republic

**Keywords:** bacterial pathogenesis, *Bordetella bronchiseptica*, *Bordetella pertussis*, mass spectrometry (MS), protein processing, serine protease

## Abstract

Filamentous hemagglutinin (FHA) mediates adherence and plays an important role in lower respiratory tract infections by pathogenic *Bordetellae*. The mature FHA proteins of *B. pertussis* (Bp‐FHA) and the *B. bronchiseptica* (Bb‐FHA) are generated by processing of the respective FhaB precursors by the autotransporter subtilisin‐type protease SphB1. We have used bottom‐up proteomics with differential ^16^O/^18^O labeling and show that despite high‐sequence conservation of the corresponding FhaB segments, the mature Bp‐FHA (~ 230 kDa) and Bb‐FHA (~ 243 kDa) proteins are processed at different sites of FhaB, after the Ala‐2348 and Lys‐2479 residues, respectively. Moreover, protease surface accessibility probing by on‐column (on‐line) digestion of the Bp‐FHA and Bb‐FHA proteins yielded different peptide patterns, revealing structural differences in the N‐terminal and C‐terminal domains of the Bp‐FHA and Bb‐FHA proteins. These data indicate specific structural variations between the highly homologous FHA proteins.

**Abbreviations**
Bb‐FHA: *B. bronchiseptica* filamentous hemagglutinin
Bp‐FHA: *B. pertussis* filamentous hemagglutinin
ESI‐FT‐ICR MS: electrospray ionization Fourier transform ion cyclotron resonance mass spectrometry
FHA: filamentous hemagglutinin
HDX: hydrogen‐deuterium exchange
LC‐MS/MS: liquid chromatography–tandem mass spectrometry

The three classical species of Gram‐negative *Bordetellae* cause respiratory infections in mammals. While *B. bronchiseptica* colonizes the nasopharynx and trachea of a broad range of mammalian hosts, such as rodents or dogs, *B. pertussis* is a strictly human pathogen that causes the highly contagious respiratory disease called whooping cough or pertussis. *B. parapertussis* typically infects ovines but human‐adapted strains of *B. parapertussis*_*hu*_ account for up to 20% of human whooping cough cases 1.

Introduction in the 1950s of whole‐cell pertussis (wP) vaccines, composed of killed *B. pertussis* cells, led to a dramatic decrease in pertussis‐related mortality and incidence of the disease 2. Safety concerns, however, led later to the replacement of the wP vaccine with the less reactogenic acellular pertussis component vaccines (aP). The latter are composed of one to five purified pertussis proteins, including chemically inactivated pertussis toxin (PT), filamentous hemagglutinin (FHA), pertactin (PRN), and/or fimbriae of serotype 2 or 3 (FIM2, FIM3). Recent epidemiologic data show a steep increase in pertussis incidence in adolescents and adults, which is linked to the switch from the use of wP to aP vaccines in developed countries in the late 1990s 3. While being effective in preventing clinical pertussis disease in infants, the aP vaccines appear to confer a rapidly waning protection and do not prevent bacterial colonization and transmission of the pathogen in aP‐vaccinated populations 4, 5, 6.

The mature *B. pertussis* FHA is included in all but one of the used aP vaccines, as FHA was proposed to play an important role in bacterial adhesion and invasion of host epithelial and phagocytic cells 7. It is a hairpin‐shaped molecule (50 nm in length and approximately 4 nm in width) consisting predominantly of tandem repetitive β‐strands arranged into a right‐handed parallel β‐helix 8. Mature FHA or its FhaB precursor was found to mediate bacterial adherence to a wide range of cell lines *in vitro* and FhaB appears to play a role in colonization of the lower respiratory tract in rodents, such as rats and mice 9, 10, 11. Four different functional domains (heparin‐binding, carbohydrate recognition, Arg‐Gly‐Asp motif, and mature C‐terminal domain) of FHA were identified and implicated in interaction of mature FHA with eukaryotic cells *in vitro*. However, the roles played by these domains in *Bordetella* infections *in vivo* are poorly defined and remain controversial 12. In addition to a role in bacterial adherence, the FHA protein was proposed to exert immunomodulatory signaling, inducing secretion of tolerogenic IL‐10 by dendritic cells 13, 14. However, this was recently shown to be due contamination of FHA preparations by endotoxin‐associated TLR2 ligands 15. Moreover, FHA was also reported to interact with the adenylate cyclase toxin, an important *Bordetella* virulence factor 16, 17.

Filamentous hemagglutinin of *B. pertussis* is synthesized as a 367‐kDa precursor (FhaB) that is exported across the cytoplasmic membrane by the general Sec system, using an unusually long N‐terminal signal peptide comprising 71 amino acid residues. The signal peptide of FhaB contains two cysteines (Cys_24_ and Cys_31_) that are necessary for post‐translational cyclization of the N‐terminal glutamine residue (Gln‐72) of processed FhaB to a cyclic pyroglutamyl residue 18. After removal of the signal sequence, the FhaB protein is secreted across the outer bacterial membrane by a two‐partner secretion (TPS) pathway 19. The N‐terminal ‘TPS domain’ of FhaB, comprising 245 residues, initiates export across the outer membrane by interacting with the periplasmic polypeptide transport associated (POTRA) domain of FhaC, the outer membrane component of the TPS secretion pathway 20. Translocation of FhaB proceeds in an N‐ to C‐terminal direction, where the N terminus forms an extended hairpin through the FhaC channel and the C terminus gradually folds into a β‐helix, as it emerges on the cell surface 21. The translocated portion of FhaB is then eventually processed by the outer membrane‐associated protease SphB1 to a 230‐kDa mature FHA protein. The ~ 1300 residue‐long C‐terminal fragment of FhaB, called the prodomain, was recently proposed to serve as an intramolecular chaperone and appears to be rapidly degraded in bacterial periplasm 22, 23, 24.

SphB1 is a surface‐exposed autotransporter protein that harbors a subtilisin‐type serine protease domain. It was proposed to cleave FhaB of *B. pertussis* within the PLFETRIKFID sequence (residues 2362–2372), but the cleavage site was not identified 25. Moreover, in SphB1‐deficient (*ΔsphB1*) strains, the FhaB precursor can still be processed to a larger FHA* protein by another, as yet unknown, protease 21, 23, 24.

Therefore, we used differential ^16^O/^18^O labeling and proteomics to identify the C‐terminal residues of FHA proteins purified from culture supernatants of wild‐type *B. pertussis* and *B. bronchiseptica* strains. The results show that despite high‐sequence conservation of the processed segments, the FhaB proteins from the two species are processed at different sites. Furthermore, the N‐ and C‐terminal domains of the two resulting FHA proteins exhibit a different surface accessibility to proteolytic cleavage.

## Material and methods

### Bacterial strains and growth conditions

*Bordetella pertussis* Tohama I and *Bordetella bronchiseptica* RB50 cells were grown at 37 °C on Bordet–Gengou agar (BG) supplemented with 15% defibrinated sheep blood. For liquid cultures, the bacteria were grown in Stainer–Scholte (SS) medium supplemented with 1 mg·mL^−1^ (2,6‐O‐dimethyl)‐β‐cyclodextrin at 37 °C.

### Purification of FHA

*Bordetella cells* were grown in 50 mL of SS medium for 8 h at 37 °C, diluted in fresh SS medium (200 mL and 1 l for *B. pertussis* and *B. bronchiseptica*, respectively) to OD_600_=0.2 and cultivated for 36 or 14 h for *B. pertussis* or *B. bronchiseptica*, respectively, using a rotary shaker (160 r.p.m.) at 37 °C. The cells were spun down at 14 000 ***g*** for 25 min at 4 °C, and the supernatants were filtered through a 0.2‐μm TPP Rapid Filtermax Vacuum Filtration system. The filtrates were loaded onto 5 mL bed volume of Cellufine sulfate (JNC Corporation, Japan) equilibrated with 10 mm phosphate buffer, pH 7.6 (PB), extensively washed with PB, and purified FHA proteins were eluted with PB supplemented with 700 mm NaCl. The purification procedure was performed at 4 °C. The purity of proteins was determined by sodium dodecyl sulfate–polyacrylamide gel electrophoresis (SDS/PAGE), and the protein concentrations were determined by Bradford assay using bovine serum albumin as standard. Due to low yields, *B. bronchiseptica* FHA was concentrated by precipitation with acetone (4 : 1, v/v) at −20 °C for 12 h and collected by centrifugation at 16 000 ***g*** for 10 min at 4 °C. Protein pellets were reconstituted in phosphate‐buffered saline (PBS) or PBS supplemented with 4 m urea (for on‐line digestion).

### Protein digest and ^18^O stable isotope labeling

Purified FHA proteins were separated on 5% SDS/PAGE gel and stained with Coomassie brilliant blue R‐250. Protein bands were excised from the gel, cut into small pieces and destained by sonication in 200 μL of Tris/HCl (pH 8.2) and 200 μL of acetonitrile (ACN). After complete destaining, the gel pieces were rinsed with 200 μL of ACN for 5 min, the liquid was discarded, and gel pieces were washed with 200 μL of H_2_O. Finally, the gel was washed by 200 μL of H_2_O/ACN (1 : 1) and dried under vacuum. Next, the gel was rehydrated in 50 μL of 10% ACN in 25 mm N‐ethyl morpholine acetate buffer (pH 8.2) containing the protease. The buffer was prepared either with normal water, or doubly concentrated buffer was diluted 1 : 1 with H_2_^18^O. Proteins were digested at 37 °C overnight, and the proteases used were as follows: trypsin gold (enzyme‐to‐substrate ratio [w/w] of 1 : 75), LysC, and AspN (enzyme‐to‐substrate ratio [w/w] of 1 : 50 for both). After digestion, the peptides were extracted with 100 μL of 80% ACN, 0.1% trifluoroacetic acid (TFA), dried via vacuum centrifugation, and solubilized in 100 μL of 10% ACN and 0.1% TFA. Alternatively, 50 μg samples of purified FHA was dried, solubilized in 50 mm ammonium bicarbonate buffer (pH 8.2), and digested using the same proteases as described above. In‐solution digestion was carried out for 6 h. Following digestion, samples were dried and reconstituted as above. Samples from in‐gel and in‐solution digestion were next desalted by peptide MacroTrap (Optimize Technologies) and eluted with 150 μL of 80% ACN, 0.1% TFA. Desalted peptides were dried via vacuum centrifugation and dissolved in 30 μL of 5% ACN, 0.1% TFA (v/v) prior the LC‐MS/MS analysis.

### Mass spectrometry

For LC‐MS/MS analyses, a capillary HPLC system (1200, Agilent Technologies, Germany) connected to an ESI source of the FT‐ICR mass spectrometer (15T, SolariX XR, Bruker) was used. Peptides were separated on analytical reverse phase column (MAGIC C18 AQ, 0.2 × 150 mm, Michrom Bioresources) and separated by following gradient: 1–10% *B* in 1 min, 10–40% *B* in 50 min, where solvent *A* was 0.2% formic acid, 2.5% ACN, and 2.5% isopropanol, and solvent *B* was 0.16% formic acid in 90% ACN and 5% isopropanol. The flow rate was 4 μL·min^−1^. ESI‐FT‐ICR MS was calibrated externally using arginine clusters resulting in a mass accuracy below 2 p.p.m. For peptide, mapping instrument was operated in data‐dependent mode, where each MS scan was followed by up to five MS/MS collision‐induced fragmentations of the most intense ions.

### H/D‐like mapping of FHA using immobilized endopeptidase under denaturing conditions

Digestion of FHA, with immobilized porcine pepsin A, aspergillopepsin, or rhizopuspepsin under HDX compatible conditions, was performed as described previously 26. Briefly, the system consisted of injection and switching valves mounted with immobilized protease column, trap column (peptide MicroTrap, Optimized Technologies), and analytical column (Jupiter C18, 0.5 × 50 mm, 5 μm, 300 Å, Phenomenex), with all components immersed in an ice‐water bath. Digestion and desalting (4 min) were driven by a Shimadzu LC20‐AD pump isocratically delivering 0.4% formic acid at a flow rate of 100–200 μL·min^−1^ depending on the protease column used. Gradient separation on the analytical column was carried out by an HPLC system (Agilent Technologies 1200) running at a flow rate of 15 μL·min^−1^ Gradient elution from 5% B to 35% B in 40 min, followed by elution with 95% B, was used for separation. Solvents used were A: 0.4% formic acid and 2% ACN; and solvent B: 0.4% formic acid in 95% ACN. The outlet of the analytical column was directly connected to an electrospray ionization (ESI) source of 15T FT‐ICR mass spectrometer (Bruker Daltonics). The purified Bp‐FHA or Bb‐FHA (300 pmol) was diluted in 0.5 m glycine/HCl buffer (pH 2.3) and injected into the column system. Alternatively, Bp‐FHA, diluted 1 : 1 with 8 m urea (to give a final urea concentration of 4 m), or Bb‐FHA, resuspended in PBS containing 4 m urea, was incubated for 30 min at 50 °C before the mixture was diluted 1 : 1 with 0.5 m glycine/HCl buffer (pH 2.3) and immediately injected into the chromatography system.

### Data processing

Data processing was performed using Data Analysis 4.1 (Bruker Daltonics). Peak picking was carried out by FTMS and SNAP algorithms, and two mascot generic files were created for each analysis. Data from the unlabeled samples (specific protease digestion) and from on‐line aspartic protease digestion were searched using local MASCOT server (MatrixScience) against a single protein database containing the sequence of FHA from *B. pertussis* or *B. bronchiseptica* with no‐enzyme specificity. Peptide tolerance was set to 10 p.p.m. and fragment ion tolerance to 0.05 Da. Identified C‐terminal peptides of FHA proteins were manually searched in the ^18^O labeled samples. The mass spectrometry proteomics data have been deposited to the ProteomeXchange Consortium via the PRIDE 27 partner repository with the dataset identifier PXD008664 and 10.6019/PXD008664.

## Results

### Purification of FHA proteins

Despite use of Bp‐FHA in aP vaccines for two decades, the exact C‐terminal sequence of FHA remained unknown. To identify the C‐terminal residues of FHA of *B. pertussis* and of *B. bronchiseptica,* we have purified the mature forms of the two proteins from culture supernatants using a single‐step affinity chromatography on Cellufine sulfate. SDS/PAGE analysis revealed that both *B. pertussis* (Bp‐FHA) and *B. bronchiseptica* (Bb‐FHA) FHA preparations contained the mature and the truncated forms of FHA 25, which migrated as double bands of >250 kDa (Fig. 1). Unlike the Bp‐FHA preparation, which was almost homogenous, the Bb‐FHA preparation contained proteolytic fragments (~ 130, 100 and 75 kDa) that were recognized by a polyclonal anti‐FHA antibody (data not shown). This likely reflected the difficulty to purify Bb‐FHA, which was obtained in about 20 times lower yields despite the use of five times larger volumes of culture supernatants. Indeed, *B. bronchiseptica* was reported to release much less FHA than *B. pertussis* 28. The lower yield of Bb‐FHA might further reflect a lower affinity for the Cellufine sulfate resin, as the heparin‐binding domain sequences of Bb‐FHA and Bp‐FHA differ importantly.

**Figure 1:** The SDS/PAGE analysis of FHA preparations purified from culture supernatants of *B.pertussis* (Bp‐FHA) and *B.bronchiseptica* (Bb‐FHA). The mature (FHA) and alternatively processed (FHA_1_) forms of FHA are indicated.

### Identification of the C‐terminal residue of FHA

To identify the C‐terminal residues of the purified proteins, the bands corresponding to mature (FHA) and truncated (FHA_1_) forms of the FHA proteins were excised from the SDS/PAGE gels and digested with trypsin, AspN, or LysC proteases. In parallel, the Bp‐FHA and Bb‐FHA preparations were digested in solution and the resulting peptides were analyzed by LC‐MS/MS followed by MASCOT search. This yielded 94% and 96% coverage of the protein sequence of mature Bp‐FHA and Bb‐FHA, respectively (PRIDE Archive, project accession: PXD008664). The C‐terminal peptides of FHA proteins were identified as peptides with masses that did not match the highly specific cleavage pattern of the used proteases (X‐↓‐Asp/Glu for AspN; Lys‐↓‐X for LysC; and Arg/Lys‐↓‐X for trypsin). The C‐terminal peptides of Bp‐FHA_1_ and Bb‐FHA_1_ were further identified by peptide mapping of the in‐gel digested FHA_1_ bands (Fig. 1), as summarized in Table 1.

**Table 1:** The C‐terminal peptides of FHA and FHA_1_ proteins based on in‐gel and in‐solution digestions

		Protease	Peptide position	Peptide sequence	M_monoisotopic_ (calculated)	M_monoisotopic_ (experimental)	Error (Δ p.p.m.)
*Bordetella pertussis*	FHA	AspN	2335–2348	G.DQPVVAVGLEQPVA.T	1420.7562	1420.7509	4
		trypsin	2300–2348	R.NAQVADAGLAGPSAVAAPAVGAADVGVEPVTGDQVDQPVVAVGLEQPVA.T	4546.3192	4546.3249	1
	FHA_1_	AspN	2214–2228	R.DVGLEKRLDIDDALA.A	1641.8573	1641.8496	5
		LysC	2220–2228	K.RLDIDDALA.A	1000.5189	1000.5251	6
*Bordetella bronchiseptica*	FHA	AspN	2446–2479	D.QPVVAVGLEQPAAAVRVAPPAVALPRPLFETRIK.F	3560.0718	3560.0566	5
	FHA_1_	AspN	2335–2347	D.DALAAVLVNPHIF.T	1378.7608	1378.7514	7
		trypsin	2331–2347	R.LDIDDALAAVLVNPHIF.T	1834.9828	1834.9818	1

The C‐terminal residue of Bp‐FHA was identified as Ala_2348_, based on detection of two peptides that partially violated the expected cleavage pattern, namely the AspN peptide _2335_DQPVVAVGLEQPVA_2348_ and the tryptic peptide _2300_NAQVADAGLAGPSAVAAPAVGAADVGVEPVTGDQVDQPVVAVGLEQPVA_2348_. The N termini of both peptides complied with the expected cleavage rules (X‐↓‐Asp for AspN and Arg‐↓‐X for trypsin) but the C‐terminal Ala_2348_ residue, followed by Thr_2349_ in FhaB sequence, did not, as neither AspN nor trypsin would cleave an Ala.Thr peptide bond. Similarly, the C terminus of Bp‐FHA_1_ was identified as Ala_2228_, based on detection of the LysC peptide _2220_RLDIDDALA_2228_ and of the AspN peptide _2214_DVGLEKRLDIDDALA_2228_. The N termini of these peptides complied well with LysC (Arg/Lys‐↓‐X) and AspN (X‐↓‐Asp) cleavage rules, while the C‐terminal Ala_2228_ residue (followed Ala_2229_ in FhaB sequence) could not result from cleavage of an Ala.Ala bond by LysC or AspN.

It should be noted that the _2214_DVGLEKRLDIDDALA_2228_ peptide contains three internal aspartate residues (D) that are possible targets for AspN cleavage, while the _2222_DIDDALA_2228_, _2224_DDALA_2228,_ and _2225_DALA_2228_ fragments were not detected. This can be understood, as the tetra‐ and penta‐peptides were too small to be trapped on the desalting column and were thus not detected by MS/MS. Moreover, AspN is rather inefficient in cutting of D‐D bonds and in complete processing of all the possible cleavage sites 29.

The C‐terminal residue of Bb‐FHA could be identified only tentatively, as Lys_2479_ residue of _2446_QPVVAVGLEQPAAAVRVAPPAVALPRPLFETRIK_2479_. This was the most C terminally located peptide detected in the AspN‐generated digests of Bb‐FHA. The N‐terminal residue of this peptide could have resulted from an unspecific AspN‐mediated cleavage on the N‐terminal side of Gln_2446_, but AspN was unlikely to have cleaved at the N‐terminal side of the Phe_2480_ residue, which follows Lys_2479_ in Bb‐FHA protein. Regrettably, no other peptides allowing confirmation of the identity of the C‐terminal residue of Bb‐FHA were detected.

In contrast, the C‐terminal residue of Bb‐FHA_1_ was unambiguously identified by detection of the _2335_DALAAVLVNPHIF_2347_ and _2331_LDIDDALAAVLVNPHIF_2347_ peptides in the AspN and tryptic digests of Bb‐FHA_1_. Neither AspN, nor trypsin would cleave the _2347_Phe.Thr_2348_ bond, while AspN and trypsin would generate the Asp_2335_ and Leu_2331_ N termini, respectively.

Apart from the peptides covering the analyzed Bp‐FHA and Bb‐FHA proteins, the detailed analysis of MS spectra revealed that both FHA preparations contained also peptides originating from *Bordetellae* proteins other than FHA. As shown in Table 2, four and five additional proteins were identified as contaminants of the Bp‐FHA and Bb‐FHA preparations. Bp‐FHA contained traces of the putative phospholipid‐binding protein MlaC, of the toluene tolerance protein Ttg2D, and of the S4 and S5 subunits of pertussis toxin. The Bb‐FHA preparation was contaminated by adenylate cyclase toxin (CyaA), the SphB1 protease, and the Bsp22, BteA, and BopD proteins secreted by the type III secretion system.

**Table 2:** The overall protein content in the Bp‐FHA and Bb‐FHA preparations

	Protein	MW (kDa)	Isoelectric point (pI)
Bp‐FHA	Filamentous hemagglutinin	367	9.2
	Pertussis toxin subunit 4	14	9.2
	Pertussis toxin subunit 5	13	5.4
	Toluene tolerance protein Ttg2D	20	9.2
	Probable phospholipid‐binding protein mlaC	21	9.2
Bb‐FHA	Filamentous hemagglutinin	372	8.7
	Adenylate cyclase toxin	178	4.4
	SphB1 protease	87	9.7
	T3SS protein BopD	32	6.4
	T3SS protein Bsp22	22	7.2
	T3SS protein BteA	69	5.0

To corroborate the identification of the C‐terminal residues of Bp‐FHA and Bb‐FHA proteins, we performed differential stable ^18^O isotope labeling. The method is based on protease‐catalyzed ^18^O replacement of two ^16^O atoms on the carboxyl of a newly liberated C‐terminal residue of a peptide that is generated by proteolytic cleavage of a protein in the presence of isotopic water (H_2_^18^O) 30. As the carboxyl of the preexisting C‐terminal residue of the digested protein remains unlabeled, the resulting mass difference between the labeled and the unlabeled peptide ions permits the identification of the peptide that contains the C‐terminal residue of the given protein.

As shown in Fig. 2, the isotope envelopes of the _2335_DQPVVAVGLEQPVA_2348_ and _2214_DVGLEKRLDIDDALA_2228_ peptide peaks in the ^18^O‐labeled AspN digests of the Bp‐FHA and of the Bp‐FHA_1_ proteins were identical to that observed for the same peptides in nonlabeled digests. The same was true for the _2446_QPVVAVGLEQPAAAVRVAPPAVALPRPLFETRIK_2479_ and _2335_DALAAVLNPHIF_2347_ peptides derived from Bb‐FHA and Bb‐FHA_1_ (Fig. 2). In contrast, the isotope envelopes of all other peptides in the ^18^O‐labeled AspN digests of Bp‐FHA/Bp‐FHA_1_ and Bb‐FHA/Bb‐FHA_1_ proteins exhibited the expected shifts to ‘double peaks’. These comprised strikingly enhanced intensities of the monoisotopic masses of the ^18^O‐labeled peptides, as documented in Fig. 2 for the internal _2279_DALASLASL_2288_ and _1086_DLQAGRSMTLGTVDTTG_1102_ peptides from the Bp‐FHA and Bb‐FHA proteins. These data thus fully confirmed that Ala_2348_ and Ala_2228_ were the C‐terminal residues of Bp‐FHA and of Bp‐FHA_1_, while Lys_2479_ and Phe_2347_ were the C‐terminal residues of Bb‐FHA and of Bb‐FHA_1_, respectively.

**Figure 2:** Isotope profiles of the C‐terminal peptides of FHA and FHA_1_ after enzymatic digestion of Bp‐FHA (upper panel) and Bb‐FHA (lower panel) with AspN in the presence of normal H_2_O (unlabeled) and 50% ^18^O water (^18^O‐labeled).

### Mapping of FHA surface accessibility using immobilized endopeptidase columns

To gain insight into the specific sequence‐structure relationships of the Bp‐FHA and Bb‐FHA proteins, we performed an on‐line digestion of the two proteins on immobilized acid protease columns connected to an LC‐MS/MS analyzer. This instrumental setup comprises a continuous workflow system that is commonly employed for analysis of protein hydrogen/deuterium exchange (HDX) by mass spectrometry 26. The main advantage of this protocol is the rapidity of digestion and the absence of sample handling. This minimizes sample loss and unwanted protein modifications that may occur during lengthy digestions in typical proteomic protocols.

Initial experiments with on‐line digestion of Bp‐FHA on an immobilized pepsin column at low pH (2.3) gave low peptide yields with sequence coverage of only 21% (data not shown). Remarkably, the recovered peptides predominantly originated from the C terminus of the mature Bp‐FHA protein (residues 1600–2350), indicating that the C‐terminal segment of Bp‐FHA is much more susceptible to protease digestion than its N‐terminal segment that exhibits a compact parallel β‐helical fold 8, 29. To increase the sequence coverage of the N‐terminal portion of FHA 19, the on‐line digestion was performed in the presence of denaturing agents, such as 3 m guanidine chloride or 4 m urea. These conditions usually do not denature proteins, but induce a partial destabilization of compact protein folds. Moreover, such concentrations of denaturing agents do not affect the cleavage efficiency of the immobilized proteases 26. Different protease columns (pepsin, nepenthesin‐1, aspergillopepsin, and rhizopuspepsin) along with different times and temperatures of digestion were also tested. Preliminary experiments showed that the best results were obtained on columns with immobilized pepsin proteases and operated and at flow rates of 100–200 μL·min^−1^ at 50 °C.

The on‐line digest peptide map acquired under such conditions covered near completely the sequence of Bp‐FHA, starting from the N‐terminal pyroglutamate residue 72, up to the C‐terminal Ala_2348_ residue (Fig. 3). In contrast, the sequence coverage of the on‐line digest of Bb‐FHA was less complete (Fig. 3). The on‐line digestion was performed for a limited time under semidenaturing conditions, using proteases that mostly cleave C terminally to frequently occurring small hydrophobic residues. Therefore, the numbers of generated unique peptides, comprising a given residue of the FHA protein, reflect the accessibility of the corresponding segment to proteolytic cleavage and the compactness of its structure. The quantitative analysis of the peptide maps revealed a striking difference in the overall distribution of unique peptides that were generated by on‐line digestion of the Bp‐FHA and Bb‐FHA proteins (Fig. 3). Irrespectively of the protease used, importantly higher number of unique peptides was recovered from the C‐terminal segment of Bp‐FHA, than from its N‐terminal segment, thus indicating a loosened conformation of the C‐terminal segment of Bp‐FHA. In contrast, the C‐terminal segment of Bb‐FHA yielded disproportionally low numbers of unique peptides, which is indicative of a tightly packed structure. In contrast, substantially higher numbers of unique peptides were generated from the N‐terminal segment of Bb‐FHA, indicating its loosened structure (Fig. 3). This would go well with the fact that the N‐terminal segment of Bb‐FHA is about 131 residues longer than the corresponding segment of Bp‐FHA. On the other hand, the C‐terminal processing of the Bp‐FHA and Bb‐FHA proteins occurred at sites 21 residues apart within a segment of very high‐sequence homology of the Bp‐FHA and Bb‐FHA proteins (Fig. 4).

**Figure 3:** Surface accessibility of Bp‐FHA and Bb‐FHA probed by on‐column (on‐line) digestion. The FHA proteins were incubated in the presence of 4 m urea at 50 °C for 30 min and loaded on immobilized protease columns directly coupled to LC‐MS/MS analyzer. Frequency of the appearance of individual residues in the covered sequence is plotted as the number of unique peptides against the protein sequence. The data represent the aggregate result obtained from the on‐line digests using rhizopuspepsin, pepsin A, and aspergillopepsin columns.

**Figure 4:** Schematic representation of the C termini of FHA proteins. FHA is encoded by the *fhaB* gene and translated as a FhaB precursor polypeptide (3590 residues in *Bordetella pertussis* and 3710 residues in *Bordetella bronchiseptica*), containing the N‐terminal signal peptide (71 residues) that is removed during translocation of FhaB across the cytoplasmic membrane. FhaB is then exported from the periplasmic space through the outer membrane and processed in SphB1‐dependent manner, yielding mature [C terminus at position 2348 (Bp‐FHA) or 2479 (Bb‐FHA)] or truncated [C terminus at position 2228 (Bp‐FHA) or 2347 (Bb‐FHA)] variant of FHA protruding on the cell surface. The C‐terminal FhaB prodomain (130 kDa) remains in the periplasm, and it is rapidly degraded. The C‐terminal peptides identified by LC‐MS/MS approaches after digestion with AspN (blue), LysC (red), trypsin (green), rhizopuspepsin (orange), and (aspergillo)pepsin (magenta) are indicated over the Bp‐FHA and Bb‐FHA protein sequences aligned based on sequence homology.

## Discussion

Release of many proteins and peptides from eukaryotic and prokaryotic cells involves proteolytic maturation of the secreted protein precursors. Production of the mature FHA protein of *Bordetella pertussis* involves processing of the 367‐kDa FhaB precursor, from which the bacterial surface‐anchored autotransporter subtilisin‐type protease SphB1 removes the 130‐kDa C‐terminal prodomain 23, 31, 32. Here, we have defined the C‐terminal residues of the mature and alternatively processed forms of FHA from the closely related *B. pertussis* and *B. bronchiseptica* species.

Up to now, the C terminus of the mature FHA protein could not be accurately identified and it was only estimated by mass determination of purified *B. pertussis* FHA. The reported MALDI‐TOF analysis indicated that mature Bp‐FHA may arise from FhaB processing within the PLFETRIKFID sequence between residues 2362 and 2372 25. By analogy, processing of Bb‐FHA was predicted to occur between residues 2472 and 2482 of Bb‐FhaB. However, insufficient accuracy of mass determination of the 230‐kDa protein by MALDI‐TOF MS did not permit identification of its C‐terminal residue. The here‐employed digest‐based peptide mapping by high‐resolution FT‐ICR‐MS, combined with postdigestion ^18^O‐labeling analysis, yielded unambiguous identification of the C‐terminal residues of the various forms of the FHA protein (Fig. 4). Firstly, the C‐terminal residues of peptides that did not match the cleavage specificity of the used proteases indicated that the Ala_2348_ and Ala_2228_ were the *bona fide* C‐terminal residues of the mature Bp‐FHA/Bp‐FHA_1_ proteins. The Lys_2479_ and Phe_2347_ residues were then identified as the respective C‐terminal residues of the Bb‐FHA/Bb‐FHA_1_ proteins. Indeed, the molecular masses of peptides comprising these residues remained unchanged upon postdigestion ^18^O‐exchange labeling of the carboxyls of the C‐terminal residues of peptides that were newly generated by *in vitro* protease digestion in H_2_^18^O. This confirmed the correct assignment of the C‐terminal residues.

Mazar and Cotter (2006) have previously shown that the SphB1 protease is involved in proteolytic maturation of FhaB to FHA and FHA_1_ both in *B. pertussis* and in *B. bronchiseptica*. Moreover, the processed regions of the FhaB precursors from the two species exhibit a very high degree of sequence identity (Fig. 4) and the SphB1 proteases of the two species are themselves identical to 98%. It is, therefore, intriguing that processing of the FhaB proteins from the two species was found to occur at quite different sites located 21 residues apart within the same highly conserved segment of FhaB. Moreover, the processing step involved cleavage of peptide bonds between rather different pairs of residues. The bond between a small hydrophobic Ala_2348_ and a small hydrophilic Thr_2349_ residue was cleaved in Bp‐FhaB, while processing of the Bb‐FhaB protein resulted from cleavage of the bond between a positively charged Lys_2479_ and a bulky aromatic Phe_2480_ residue. As a result, the C‐terminal segment of the mature Bb‐FHA is extended by 21 residues, compared to mature Bp‐FHA. Similarly, the C‐terminal sequences of Bp‐FHA_1_ and Bb‐FHA_1_ differ by 9 residues.

Albeit unlikely, it cannot be excluded that upon SphB1‐mediated cleavage the C termini of FHA may be further processed by some other secreted bacterial proteases. Alternatively, these unexpected results may indicate that the substrate specificities of the highly conserved SphB1 proteases of the two bacterial species may differ. The SphB1 protease, indeed, belongs to a superfamily of subtilisin‐like proteases that possess rather broad substrate specificity. This is largely determined by interactions of the P4‐P1 residue side chains in the binding pocket of the enzyme, which enables the cleavage of peptide bonds on the C‐side of aliphatic or aromatic amino acid residues 33. A closer look on the P4‐P1 residues of Bp‐FHA (QPVA_2348_) and Bp‐FHA_1_ (DALA_2228_) reveals a certain analogy between their C‐terminal sequences, in terms of side chain properties, indicating that Bp‐FhaB is processed by SphB1 with a defined substrate specificity. In contrast, the C‐terminal sequences of Bb‐FHA (TRIK_2479_) and Bb‐FHA_1_ (PHIF_2347_) are rather distinct and do not appear to share any similarity, even though the C‐terminal residue of Bb‐FHA_1_ complies with the substrate specificity of subtilisin‐like proteases. However, the C‐terminal Lys_2479_ residue of Bb‐FHA does not match the substrate specificity of a subtilisin type of protease. It thus remains to be determined if the Bb‐SphB1 has a broader substrate specificity than Bp‐SphB1, or another as yet unknown protease participates in the final processing of the Bb‐FhaB precursor.

Even though the Bp‐FHA and Bb‐FHA proteins are highly homologous (90% identity) and appear to be functionally interchangeable between *B. pertussis* and *B. bronchiseptica* 34, our data show that the C termini of mature FHA proteins differ by 21 amino acid residues. The here observed difference in the processing and protease susceptibility of the C‐terminal segments of the two proteins is intriguing, as the mature C‐terminal domain of FHA was proposed to play an important role in adherence and virulence of *Bordetellae* 11, 24, 31, 34. *B. pertussis* is a fully human‐adapted pathogen, while *B. bronchiseptica* infects a broad variety of mammals. It will, hence, be important to determine whether the difference in FhaB processing in the two bacterial species plays a role in the biological activity of mature FHA proteins.

## Author contributions

DJ measured and analyzed the data, PM performed and evaluated the on‐line digests, LB and PS designed the project, and LB, DJ, and PS wrote the manuscript.
